The article "Effects of an Adenosine A2A Receptor Antagonist on Striatal Dopamine D2-Type Receptor Availability: A Randomized Control Study Using Positron Emission Tomography" was published in 2021. Journal: Front Neurosci.

# Effects of an Adenosine A_2A_ Receptor Antagonist on Striatal Dopamine D2-Type Receptor Availability: A Randomized Control Study Using Positron Emission Tomography

**DOI:** 10.3389/fnins.2021.729153

**Published:** 2021-09-13

**Authors:** Kyoji Okita, Koichi Kato, Yoko Shigemoto, Noriko Sato, Toshihiko Matsumoto, Hiroshi Matsuda

**Affiliations:** ^1^Integrative Brain Imaging Center, National Center of Neurology and Psychiatry, Tokyo, Japan; ^2^Department of Psychiatry, Center Hospital, National Center of Neurology and Psychiatry, Tokyo, Japan; ^3^Department of Drug Dependence Research, National Institute of Mental Health, National Center of Neurology and Psychiatry, Tokyo, Japan; ^4^Department of Radiology, Center Hospital, National Center of Neurology and Psychiatry, Tokyo, Japan; ^5^Cyclotron and Drug Discovery Research Center, Southern TOHOKU Research Institute for Neuroscience, Koriyama, Japan; ^6^Department of Biofunctional Imaging, Fukushima Medical University, Fukushima, Japan

**Keywords:** dopamine D2 receptors, adenosine 2A receptor, positron emission tomography, striatum, randomized control study

## Abstract

**Introduction:** Altered dopaminergic neurotransmission, especially in the functioning of dopamine D2-type receptors, is considered central to the etiology of a variety of neuropsychiatric disorders. In particular, individuals with substance use disorders have been consistently observed to exhibit lower D2-type receptor availability (quantified as binding potential; BP_ND_) using positron emission tomography (PET). Upregulation of D2-type receptor density thus may therefore provide a therapeutic effect for substance use disorders. Importantly, *in vitro* studies reveal that D2 receptors coexist with adenosine 2A (A2A) receptors to form the highest density of heteromers in the whole striatum, and there is a functional interaction between these two receptors. As such, blockade of A2A receptor’s function may prevent D2 receptor downregulation, yet no study has currently examined this hypothesis in humans.

**Methods and Analysis:** This double-blind, randomized controlled trial aims to evaluate the effect of the A2A receptor antagonist istradefylline (compared to placebo) on both dopamine D2-type receptor availability in the human brain and on neuropsychological measurements of impulsivity. It is hypothesized that istradefylline will both increase striatal D2-type BP_ND_ and improve control of impulsivity more than placebo. Forty healthy participants, aged 20–65 with no history of psychiatric or neurological disorders, will be recruited and randomized into two groups and will undergo [^11^C]raclopride PET, once before and once after administration of either 40 mg/day istradefylline or placebo for 2 weeks. Neuropsychological measurements will be administered on the same days of the PET scans.

The article "Effects of an Adenosine A2A Receptor Antagonist on Striatal Dopamine D2-Type Receptor Availability: A Randomized Control Study Using Positron Emission Tomography" was published in 2021. Journal: Front Neurosci.

**Ethics and Dissemination:** The study protocol was approved by the Certified Review Boards (CRB) of National Center of Neurology and Psychiatry (CR18-011) and prospectively registered with the Japan Registry of Clinical Trials (jRCTs031180131; https://jrct.niph.go.jp/latest-detail/jRCTs031180131). The findings of this study will be disseminated through peer reviewed scientific journals and conferences.

**Clinical Trial Registration:**www.ClinicalTrials.gov, identifier jRCTs031180131.

## Highlights

Strengths and limitations of this study:

- This double-blind randomized controlled trial is the first study to test the effects of an adenosine 2A (A2A) receptor antagonist on dopamine D2-type receptors in the living human brain.
- Both positron emission tomography with a ligand with high affinity for D2-type receptors and neuropsychological measurements will be administered both pre- and post-intervention.
- Istradefylline, the only prescription selective A2A receptor antagonist, will be used as a pharmacological intervention for 2 weeks.
- The double-blind design enables rigorous evaluation of the efficacy of A2A receptor antagonist on D2-type receptors.

## Introduction

Alterations in dopaminergic neurotransmission has been shown to play an important role in a variety of neuropsychiatric disorders such as schizophrenia (Howes and Kapur, 2009; McCutcheon et al., 2019), major depressive disorders (Belujon and Grace, 2017), Parkinson syndrome (Fahn, 2008), attention deficit/hyperactivity disorder (ADHD) (Tripp and Wickens, 2009; Kollins and Adcock, 2014), eating disorders (Wang et al., 2011; Frank, 2019), and substance use disorders (Solinas et al., 2019). With regards to the latter group of disorders, studies using positron emission tomography (PET) have repeatedly shown that compared to non-drug using healthy controls, participants who abuse drugs exhibit lower striatal dopamine D2-type receptor availability (quantified as binding potential; BP_ND_) (see reviews Volkow et al., 2009; Ashok et al., 2017; London, 2020). Moreover, in methamphetamine users, lower striatal dopamine D2-type BP_ND_ is associated both with greater impulsivity (Lee et al., 2009; Ghahremani et al., 2012; Moeller et al., 2018) and with greater drug-seeking behaviors as determined by the choosing of methamphetamine-related images in a choice task (Moeller et al., 2018).

On the basis of these findings, enhancing dopaminergic signaling through dopamine D2-type receptors may provide a therapeutic approach for substance use disorders. However, to date, no dopamine D2-type receptor agonist has provided a therapeutic effect for any addictive disorder (Verrico et al., 2013; Blum et al., 2014). Importantly, this lack of an effect may be due to the fact that such medications only stimulate D2-type receptors but do not recover D2-type receptor’s function; upregulation of D2-type receptor density may therefore provide a therapeutic effect for addictive disorders.

The article "Effects of an Adenosine A2A Receptor Antagonist on Striatal Dopamine D2-Type Receptor Availability: A Randomized Control Study Using Positron Emission Tomography" was published in 2021. Journal: Front Neurosci.

Adenosine 2A (A2A) receptors and dopamine D2-type receptors are both G protein-coupled receptors (GPCRs), and are mostly expressed on the dendritic spines of striatopallidal GABAergic neurons where they constitute the highest density of A2A receptor-D2 receptor heteromers in the whole striatum. As such, there is a strong functional interaction between these two receptors in this region (Ferre et al., 2016). For instance, selective A2A receptor antagonism suppresses D2-type receptor internalization from the membrane into the cell body of cultivated rat cells (Huang et al., 2013). On this basis, A2A receptor antagonism could prevent D2-type receptor internalization and may therefore induce upregulation of these receptors in the human living brain.

Istradefylline, a structural analog of caffeine, is a selective antagonist at the A2A receptors and is used as an add-on treatment to levodopa for Parkinson’s disease. Because its long-term safety and high tolerability has been proved (Kondo and Mizuno, 2015), istradefylline has been used for this purpose since 2013 in Japan, and since 2019 in the United States. Specifically, istradefylline partially treats the negative effects of Parkinsonism by reducing “off” periods, which are defined as those periods in which the effects of levodopa are wearing off (Tao and Liang, 2015). Although istradefylline’s selective A2A receptor antagonism may result in upregulation of D2 receptors, no study has yet examined this potential effect in the living human brain.

The main research aim of this study will be to determine whether medium-term (i.e., 2-week) administration of istradefylline can produce upregulation of dopamine D2 receptors in humans (Aim 1). It is hypothesized that participants who receive 2-week administration of istradefylline, as compared to placebo, will exhibit increased dopamine D2-type receptor BP_N__D_ as indicated by a significant group (istradefylline vs. placebo) × time (pre- vs. post-intervention) interaction (Hypothesis 1). The secondary aims will be to assess the effects of istradefylline on cognitive measures (Aim 2a), and to evaluate the extent to which any effects on cognition are related to changes in BP_ND_ (Aim 2b). Therefore, the secondary hypotheses are that istradefylline administration would improve cognitive performance more than placebo administration (as indicated by a significant group × time interaction; Hypothesis 2a), and that any effects of istradefylline administration on D2-type receptor BP_ND_ will be associated with such effects on cognitive performance (Hypothesis 2b).

The article "Effects of an Adenosine A2A Receptor Antagonist on Striatal Dopamine D2-Type Receptor Availability: A Randomized Control Study Using Positron Emission Tomography" was published in 2021. Journal: Front Neurosci.

## Methods and Analysis

### Research Design

The study is a 2-week, double-blind, placebo-controlled, randomized controlled trial that aims to determine the potential effect of istradefylline, a selective A2A receptor antagonist, on dopamine D2-type BP_ND_ within the striatum. Participants will be randomized into two groups in a between-subjects design, one in which participants will receive (40 mg/day) of istradefylline, and the other in which they will receive a placebo (see Figure 1).

**FIGURE 1:** Schematic diagram of the study.

### Participants

Forty participants, all aged 20–65 years old with no history of psychiatric or neurological disorders will be recruited for this study. Inclusion criteria are: being male, being able to comprehend Japanese and being of any race or ethnicity. Exclusion criteria include the following: smoking at least one cigarette or electronic cigarette within the past 1 year; lifetime history or current possibility of psychiatric disorder (confirmed using the Mini International Neuropsychiatric Interview; M.I.N.I.); intracranial lesion(s) as observed from the structural magnetic resonance image (MRI; see below); impairment of liver and/or renal function; HIV seropositive; positive urine-sample test for illegal drug; past history of suicidal ideation or attempt; claustrophobia or aichmophobia; metals inside the body incompatible with MRI; use of psychotropic drugs which could have an impact on dopamine D2-type BP_ND_; use of drugs that interact with CYP3A4, a major metabolizing enzyme of istradefylline; caffeine consumption greater than 400 mg/day (e.g., more than five cups of coffee per day). Female participants will not be enrolled into this current study because of the reported influence of the menstrual cycle on D2-type BP_ND_ (Wong et al., 1988; Munro et al., 2006; Czoty et al., 2009). Because the main aim of this study is to determine whether A2A receptor blockade upregulates dopamine D2 receptor in humans rather than to determine the clinical utility of such blockade in a generalized sample of participants, we decided to enroll only male participants in order to eliminate the potential confounding factor of the menstrual cycle.

#### Patient and Public Involvement

Participants were not involved in the recruitment and conduct of the study. Moreover, participants will not be involved in deciding which data and results to report. However, members of the research team may listen to input from participants during the process of deciding what to report; regardless, the final decision as to which findings to report will be made only by the scientists.

The article "Effects of an Adenosine A2A Receptor Antagonist on Striatal Dopamine D2-Type Receptor Availability: A Randomized Control Study Using Positron Emission Tomography" was published in 2021. Journal: Front Neurosci.

### Screening Visit

All aspects of this study will take place at the National Center of Neurology and Psychiatry (NCNP) in Kodaira, Tokyo, Japan. The study procedure has been reviewed and approved by the Certified Review Boards (CRBs) of NCNP. Study participants will be recruited through online methods and via print advertisement flyers distributed to public locations in Kodaira, including community centers, libraries, city halls, and schools. Potential participants will contact the research team by email or phone to be briefly screened over the phone to roughly determine eligibility; those who meet inclusion/exclusion criteria will then be invited to come into the office for further screening. At the initial in-person screening visit, participants will be given a full description of the study procedure and will be asked to read and sign the CRB-approved informed consent forms with the PI. After signing the consent form, a comprehensive baseline assessment including M.I.N.I., urine drug test, blood test and MRI scan (see below for details) will be performed for rigorous screening (see Table 1). The study physician will determine medical eligibility for the study via examination of all data acquired at the screening visit. Ineligible individuals are referred for clinical follow-up.

### Study Medication

Participants will receive either istradefylline (40 mg/day) or placebo for 2 weeks in a double-blind, between-subjects design. This dose (40 mg/day) was selected because it is the maximum dose approved in clinical practice. Both istradefylline (brand name Nourianz^®^; Kyowa Kirin, Inc., Tokyo, Japan), and placebo have been encapsulated in sufficiently opaque and colored gelatin capsules (DBcaps^®^, Lonza, Basel, Switzerland) so as not to reveal contents inside or disclose any possible difference between the two capsule types. Active medication capsules consist of two 20 mg Nourianz^®^ tablets and placebo capsules consist of two Satisfake^®^ tablets (METGREEN, Co., Ltd., Tokyo, Japan). All study capsules contain dextrose as the inert filling agent and have been brought to proper packing level in color-matched, opaque, identically sized capsules. Participants will be instructed on Day 1 to take each capsule in the morning between 6 and 8 AM (i.e., once daily) to minimize a potential risk of drug-induced insomnia (Kondo and Mizuno, 2015). As such, participants will start taking their first capsule on the following morning, and will take their final capsule on the morning of Day 15. Participants will receive email notification from the investigator team every morning to check adherence and potential side effect.

The article "Effects of an Adenosine A2A Receptor Antagonist on Striatal Dopamine D2-Type Receptor Availability: A Randomized Control Study Using Positron Emission Tomography" was published in 2021. Journal: Front Neurosci.

### Random Allocation

Participants will be randomly assigned in a 1:1 manner using a stratified block-randomization procedure with age as the stratification factor. The allocation sequence has been computer-generated and will be carried out by a study statistician who is not involved in any other study procedures in order to preserve the double-blind design. A blinded stratification list, including subject ID and age will be used to assign participants a group based on the stratification factor (i.e., active or placebo). A study pharmacist in charge will match this information to the unblinded stratification list and fills the prescription. The pharmacist is the only person who will have access to the unblinded stratification list.

### Adverse Event Reporting

An annual summary of adverse events will be submitted to the Japan Registry of Clinical Trials (jRCTs) and the CRB at NCNP. In the event that significant medical problems occur, or in the case that an investigator believes that any aspects of the study may be causing harm to participants’ health, the blinding will be unlocked and medical treatment will be provided. Significant medical problems are defined as any fatal event, any immediately life-threatening event, any permanent or substantially disabling event, any event that requires or prolongs inpatient hospitalization, any congenital anomaly, or any unexpected adverse drug experiences that have not previously been observed. The PI will promptly report all severe adverse events to the director of NCNP, the CRB of NCNP, the Pharmaceuticals and Medical Devices Agency, and the Ministry of Health, Labor and Welfare (where appropriate). A decision to unlock the blinding will be determined by the PI given the severity of the medical problem and its relevance to study medication.

### Data Monitoring

An independent review board at the Department of Clinical Epidemiology, Translational Medical Center at NCNP will perform regular monitoring over the course of the study. They will oversee the case report forms to verify that all study procedures are in compliance with approved study protocol, and to provide monitoring reports to the PI.

### Neuroimaging

#### Magnetic Resonance Image Scan

Structural MRI scans of the brain will be acquired for co-registration with PET images and definition of volumes-of-interest (VOIs). A T1-weighted scan will be acquired using a whole-brain magnetization-prepared rapid acquisition with gradient echo (MPRAGE) (TR = 1900 ms, TE = 4.38 ms, flip angle = 15, field of view = 250 × 250 × 165, 165 slices, thickness = 1 mm).

The article "Effects of an Adenosine A2A Receptor Antagonist on Striatal Dopamine D2-Type Receptor Availability: A Randomized Control Study Using Positron Emission Tomography" was published in 2021. Journal: Front Neurosci.

#### Positron Emission Tomography Scan

Positron emission tomography scans with [^11^C]raclopride, a radiotracer with selective affinity for dopamine D2-type receptors (Kohler et al., 1985) will be acquired. PET scans with [11C]raclopride will be acquired; importantly, the test-retest reliability of the scan has been shown to be good (Alakurtti et al., 2015). Participants will undergo 2 PET scan; one scan pre-intervention and a second scan 6 h after the final drug administration, both of which will begin at 1 PM local time. PET data were acquired using a Biograph TruePoint 6 PET/CT (Siemens Healthineers, Erlangen, Germany), which has a resolution full-width at half-maximum (FWHM) of 4.1 mm, and an axial field of view of 162 mm in the 3D mode. Participants will be placed in the supine position, with their head secured with a plastic band to avoid movement during the scan. After a low-dose CT scan was performed for attenuation correction, emission data will be collected for 60 min after a bolus injection of 10 mCi (±10%; range of 9–11 mCi) [^11^C]raclopride, which has a specific activity of > 1 Ci/μmol.

### Data Processing

Using the 3-dimention ordered subset expectation maximization (3D-OSEM) algorithm (Lee et al., 2014), the PET data will be reconstructed into twelve 20-s frames, sixteen 60-s frames, and ten 240-s frames (Kubota et al., 2017). FSL MCFLIRT (FMRIB Centre, Dept. Clinical Neurology, University of Oxford) will be used for motion correction (Jenkinson et al., 2002). The images will then be co-registered to the MPRAGE image using a 6-parameter, rigid-body spatial transformation (FSL FLIRT).

VOIs will be derived from individual MPRAGE images using FSL FIRST (Patenaude et al., 2011). Caudate and putamen VOIs will be combined to constitute a single striatum VOI. The cerebellum will be used as the reference region (Hall et al., 1994). A cerebellum VOI, including the hemispheres but not the vermis, will be manually created in standard space (MNI152 template) and transformed into native space with FSL FNIRT.

Time-activity data within VOIs will be extracted from PET images and imported into PMOD Kinetic Modeling (PKIN) (PMOD Technologies Ltd., Zurich). The simplified reference tissue model (SRTM), will be used to calculate BP_ND_. This method will be used because its accuracy for [11C]raclopride scans has been fully validated (Farde et al., 1989; Lammertsma and Hume, 1996; Lammertsma et al., 1996), and because this method eliminates the need for measuring the arterial input function which in turn avoids the potential risks associated with arterial cannulation. BP_ND_ will be calculated with time–activity curves from VOIs as follows: *C*_T_(*t*) = R1C_R_(*t*) + (k2 – R1k2/(1 + BP_ND_))*C*_R_(*t*) ^∗^ exp(−k2t/(1 + BP_ND_)) where *C*_T_(*t*) is the total radioactivity concentration in the striatum VOI measured by PET, R1 is the ratio of K1–K1’ (K_1_, influx rate constant for the striatum; K1’, influx rate constant for the cerebellum), *C*_R_(*t*) is the radioactivity concentration in the reference region (cerebellum), and ^∗^ denotes the convolution integral. The parameters R1, k2, and BP_ND_ in this model are estimated by a non-linear curve-fitting procedure.

The article "Effects of an Adenosine A2A Receptor Antagonist on Striatal Dopamine D2-Type Receptor Availability: A Randomized Control Study Using Positron Emission Tomography" was published in 2021. Journal: Front Neurosci.

### Neuropsychological Measurements

The following measurements will be administered starting at 10 AM on each day of PET scan (i.e., 3 h before the scan) (see Table 1).

**TABLE 1:** Schedule of enrollment and assessment.

	In-person screening session	Administration period		Post administration period
	
Day		Day 1	Day 15	Day 22
Informed consent	x			
Participant characteristics	x			
Clinical examination	x			
Mini International Neuropsychiatric Interview	x			
Blood sample test for HIV, hepatitis, liver/kidney failure	x			
MRI scan	x			
Blood pressure	x	x	x	
Height, body weight, and body composition measurement	x	x	x	
Body temperature	x	x	x	
Urine sample test (drug screen)	x	x	x	
Barratt Impulsiveness Scale		x	x	
Stop-signal task		x	x	
Monetary Choice Questionnaire		x	x	
Toronto Alexithymia Scale		x	x	
Difficulties in Emotion Regulation Scale		x	x	
Beck Depression Inventory		x	x	
Beck Anxiety Inventory		x	x	
PET scan with [11C]raclopride		x	x	
Side Effect Screen			x	x

#### Barratt Impulsiveness Scale

This 30-item self-report questionnaire assesses impulsive personality traits (Patton et al., 1995). A form of this measure that is sensitive to changes in impulsivity over time (Ghahremani et al., 2013) will be used.

#### Stop-Signal Task

On “go” trials, a series of visual stimuli are presented to prompt pressing a left or right corresponding key. On “stop” trials (i.e., 25% of all trials), a tone (i.e., a “stop-signal”), will be presented after a short delay after the “go” stimulus (this delay is termed the stop-signal delay; SSD); this “stop-signal” will indicate to the participant that they should withhold responding. The SSD is adjusted on a trial-by-trial basis according to performance. The primary dependent variable, stop-signal reaction time, is the mean difference between the SSD and the reaction time to “go” stimuli, and indicates how quickly the participant can inhibit an ongoing motor response.

#### Monetary Choice Questionnaire

Participants must select between one of two hypothetical options in 27 questions to receive a certain amount of money immediately or a larger amount later. The discrepancies between the monetary amounts and duration of the delay are varied across questions. A hyperbolic statistical function is fit to the data to estimate the individual’s point of indifference between the options. The primary dependent variable is the indifference point, or total k value, determined from the participant’s selections across the task. Scores are typically adjusted with the natural log to compensate for skew (Kirby et al., 1999).

The article "Effects of an Adenosine A2A Receptor Antagonist on Striatal Dopamine D2-Type Receptor Availability: A Randomized Control Study Using Positron Emission Tomography" was published in 2021. Journal: Front Neurosci.

#### Toronto Alexithymia Scale-20

Emotional self-awareness will be assessed using the Toronto Alexithymia Scale-20 (TAS-20; Bagby et al., 1994), a widely used questionnaire that consists of three subscales that provide scores for corresponding factors. Two of the factors assess emotional self-awareness: Factor 1: Difficulty Identifying Feelings; and Factor 2: Difficulty Describing Feelings. Factor 3 assesses Externally-Oriented Thinking. TAS-20 total score (the sum of the three subscale scores) is interpreted as follows: 0–51: no alexithymia; 52–60: possible alexithymia; 61 and above: alexithymia (Taylor et al., 1999).

#### Difficulties in Emotion Regulation Scale

Difficulties in Emotion Regulation Scale (DERS) will be administered to assess an emotion dysregulation (Gratz and Roemer, 2004). This 36-item questionnaire is divided into six-distinct subscales: Non-acceptance of Emotional Responses (NON-ACCEPT); Difficulties Engaging in Goal-Directed Behavior (GOALS); Impulse Control Difficulties (IMPULSE); Lack of Emotional Awareness (AWARE); Limited Access to Emotion Regulation Strategies (STRATEGIES); and Lack of Emotional Clarity (CLARITY). Scores on each subscale can be summed to create a total score which can range from 30 to 180; higher scores represent more difficulties in emotion regulation.

#### Beck Depression Inventory and Beck Anxiety Inventory

The Beck Depression Inventory (BDI) (Beck et al., 1996) and Beck Anxiety Inventory (BAI) (Beck et al., 1988) are self-report inventories to verify depressive and anxiety symptoms respectively. They will be employed to verify exclusion criteria and monitor potential adverse event related to drug administration.

### Data Analytic Plan

#### Power Considerations

A sample size was selected based on a power analysis that was performed previously. Eighteen subjects per group is assumed to be necessary to provide sufficient power (β > 0.8) to detect interaction effects as small as *f* = 0.2, assuming a within-subject correlation coefficient of 0.8 based on previous study (Alakurtti et al., 2015) for the repeated measures and two-sided significance of α = 0.05. Taking into account the potential drop out from the study of roughly 10% of all recruited participants, we set a sample size of *N* = 40. A previous study that aimed to show D2-type receptor upregulation in humans after completion of an exercise intervention revealed a group-by-time interaction on the dependent variable to the magnitude of *f* = 0.28 (Robertson et al., 2016). Thus, the current study appears to be powered to detect a significant effect in our main aim.

The article "Effects of an Adenosine A2A Receptor Antagonist on Striatal Dopamine D2-Type Receptor Availability: A Randomized Control Study Using Positron Emission Tomography" was published in 2021. Journal: Front Neurosci.

#### Statistical Analysis

We will use graphical and numerical summaries to screen the data for outliers and violations of model assumptions. For Aim 1, the hypothesis will be tested by evaluating the effects of treatment group (istradefylline vs. placebo), time (pre- vs. post-intervention), and the group-by-time interaction on D2-type BP_ND_ (which will be the dependent variable) using a repeated measures ANCOVA. In *post hoc* tests, the effect of time will be tested using paired *t*-tests in each group to identify the sign of any interaction effect. For Aim 2a, the hypothesis will be tested by using the same above-defined ANCOVA model but with cognitive measures as the dependent variable instead of D2-type BP_ND_. For aim 2b, partial correlation analysis will be performed to evaluate the potential associations between change in BP_ND_ and change in cognitive measures. These statistical analyses will be conducted using SPSS IBM 19 (IBM, Armonk, NY, United States).

## Discussion

A variety of psychiatric and neurological disorders are characterized by impaired dopaminergic neurotransmission through dopamine D2-type receptor. In particular, lower striatal D2-type BP_ND_ has been repeatedly observed in participants with substance use disorders when compared with healthy controls (Volkow et al., 2009; Ashok et al., 2017; London, 2020). Importantly, because such observations were made from cross-sectional studies, it may be that these findings could reflect innate biological characteristics of individuals with substance use disorders that precede the initiation of substance use. However, given that most addictive substances have been shown to induce phasic dopamine release in the human brain (Nutt et al., 2015), and because agonism of GPCRs initiates processes that are involved in the subsequent desensitization of these receptors that is associated with their downregulation (Ferguson, 2001; Tabor et al., 2017), it seems likely that accumulative substance use contributes to D2-receptor downregulation (Volkow et al., 2004). Further, *in vitro* studies using cultured cells derived from human neuroblastoma indicate that concurrent agonist stimulation of A2A receptors and D2 receptors induces coaggregation and co-internalization of those receptors into cell bodies (Hillion et al., 2002; Bartlett et al., 2005). Therefore, A2A receptor antagonists may help to upregulate D2 receptors by preventing such receptor internalization.

The article "Effects of an Adenosine A2A Receptor Antagonist on Striatal Dopamine D2-Type Receptor Availability: A Randomized Control Study Using Positron Emission Tomography" was published in 2021. Journal: Front Neurosci.

A human longitudinal PET study using the same PET ligand as we will use in this study has shown that striatal D2-type receptor availability increases after a single administration of caffeine. Because caffeine is an agonist of not only the A2A receptor subtype, but also of other subtypes of adenosine receptors; it may be that this increase in D2-type receptor availability is a consequence of controlling D2 receptor internalization by A2A receptors (Volkow et al., 2015). To date, this is the only study that has demonstrated the potential allosteric effect between A2A receptors and D2 receptors in the living human brain. However, since caffeine has an antagonistic action on any subtype of adenosine receptors (Ribeiro and Sebastiao, 2010), the results of Volkow et al. (2015) do not necessarily indicate that an A2A receptor antagonist could induce D2-type receptor upregulation. In addition, although the study design employed by Volkow et al. (2015) was a simple pre- vs. post-comparison, it would be prudent to employ a randomized control trial design to eliminate any possible evaluation biases.

Thus, the proposed study will monitor changes in striatal D2-type receptor BP_ND_ due to administration of istradefylline, a selective A2AR antagonist using a double-blind, randomized, placebo-controlled design. Importantly, our study design cannot distinguish between acute and chronic effects because the interval between the last drug administration and a final (i.e., second) scan is only 6 h. However, positive findings, positive findings from this study would have wide-ranging significance, especially for the potential treatment of a variety of neuropsychiatric disorders that are characterized by dysfunctional dopamine D2-type receptors, for many of which no pharmacological intervention has been proven effective.

## Data Availability Statement

The raw data supporting the conclusions of this article will be made available by the authors, without undue reservation.

## Ethics Statement

The studies involving human participants were reviewed and approved by Certified Review Boards of the National Center of Neurology and Psychiatry. The patients/participants provided their written informed consent to participate in this study.

## Author Contributions

All authors made a significant contribution to the conception and design of the trial protocol. KO is the PI of the study and made major contributions to the design of this trial, development of the original trial protocol and drafting of the initial manuscript.

The article "Effects of an Adenosine A2A Receptor Antagonist on Striatal Dopamine D2-Type Receptor Availability: A Randomized Control Study Using Positron Emission Tomography" was published in 2021. Journal: Front Neurosci.

## Conflict of Interest

The authors declare that the research was conducted in the absence of any commercial or financial relationships that could be construed as a potential conflict of interest.

## Publisher’s Note

All claims expressed in this article are solely those of the authors and do not necessarily represent those of their affiliated organizations, or those of the publisher, the editors and the reviewers. Any product that may be evaluated in this article, or claim that may be made by its manufacturer, is not guaranteed or endorsed by the publisher.
